The article "Febuxostat Improves Uric Acid Levels and Renal Function in Patients with Chronic Kidney Disease and Hyperuricemia: A Meta-Analysis" was published in 2022. Journal: Appl Bionics Biomech.

# Febuxostat Improves Uric Acid Levels and Renal Function in Patients with Chronic Kidney Disease and Hyperuricemia: A Meta-Analysis

**DOI:** 10.1155/2022/9704862

**Published:** 2022-07-08

**Authors:** Yanqun Zheng, Jia Sun

**Affiliations:** Nephrology Department, First People's Hospital of Linping District, Hangzhou, China

## Abstract

**Background:**

Uric acid nephropathy, also known as hyperuricemia nephropathy or gouty nephropathy, is characterized by uric acid crystal deposition and inflammatory cell infiltration. Herein, we aimed to demonstrate the role of febuxostat on uric acid levels and renal function in patients with chronic kidney disease and hyperuricemia.

**Methods:**

Eight databases included were searched for clinical randomized controlled trials. Meanwhile, the confidence interval (CI) of either relative risk or mean difference was set to 95%. Besides, the heterogeneity of the research results is tested by *I*^2^.

**Results:**

Ten studies were ultimately included in this meta-analysis. All of them were considered to be random controlled trials. 10 studies reported the serum uric acid of the test group and the control group, which was significantly lower (SMD: -146.44, 95% Cl: -195.96, -86.93, and *P* < 0.01) than the control group, EGFR (SMD: 3.21, 95% Cl: 1.17, 5.25, and *P* < 0.01), serum creatinine (SMD: -15.27, 95% Cl: -20.75, -9.79, and *P* < 0.01), serum urea nitrogen (SMD: -2.37, 95% Cl: -3.31, -1.61, and *P* < 0.01), and adverse reactions (OR: 0.74, 95% Cl: 0.32, 1.68, and *P* = 0.47).

**Conclusion:**

The results of this study suggest that febuxostat may be effective in patients with CKD with HUA, as evidenced by serum uric acid, creatinine, urea nitrogen, and EGFR. However, large sample, multicenter, low risk of bias clinical studies, as well as basic medical research, are needed.

## 1. Introduction

Hyperuricemia (HUA), commonly defined in the literature as serum uric acid (sUA) levels above 6 mg/dl [1], has a prevalence of 21% in the United States [2]. It is associated with a higher risk of high blood pressure, coronary artery disease, and stroke [3]. HUA is associated with the pathophysiology of kidney disease, making clinical research an active research interest [4, 5].

Previous meta-analyses have shown that HUA is a risk factor for the development of chronic kidney disease (CKD) and incidental kidney disease, including end-stage renal disease, albuminuria, or elevated serum creatinine [6]. Rodenbach et al. [7] conducted a 5-year cross-sectional study, and the results showed that the HUA group of CKD children had a worse prognosis than the normal serum uric acid group. It was reported that more than 70% of HUA patients suffered from different degrees of HUA. 36.3% of patients tend to have renal failure [8]. Another study showed that nearly 0.6% to 1.0% of patients with renal failure were caused by gout. A New Zealand report showed that the patients who died due to gouty nephropathy can account for 16% to 27% of the patients who died due to gout complications [9].

Febuxostat is a novel xanthine oxidase-selective inhibitor that inhibits both xanthine oxidase and xanthine dehydrogenase activities and reduces blood urate concentrations [10]. Febuxostat is mainly metabolized by the liver into inactive metabolites, which can be completely excreted from the body. Therefore, the metabolic process is less affected by renal function, and its renal toxicity is also mild. To a certain extent, it can improve renal function and reduce serum creatinine [11, 12]. Thus, we conducted a meta-analysis to examine the efficacy and safety of febuxostat in patients with CKD with HUA.

## 2. Materials and Methods

### 2.1. Eligibility Criteria

#### 2.1.1. Study Design

All randomized controlled trials (RCTs) investigating febuxostat combined with other therapies in the treatment of CKD with HUA were not limited by language or publication status.

#### 2.1.2. Research Object

This includes patients with CKD with HUA, with no recent history of drug therapy such as febuxostat and allopurinol.

#### 2.1.3. Intervention Measures

The experimental group was treated with febuxostat or febuxostat in combination with other therapies for intervention, and the control group was treated with nonfebuxostat, including allopurinol or placebo therapy. In addition, the following exclusion criteria were applied: ① nonrandomized controlled trial research literature, ② literature that did not report febuxostat as an intervention measure, ③ literature without original data or incomplete research data, ④ inconsistent outcome indicators or statistical methods, and ⑤ literature review or animal experiment research.

#### 2.1.4. Outcome Indicators

Through the review of clinical trials published in major databases and academic journals to evaluate CKD with HUA, we found that the commonly used evaluation indicators include the following: ① serum uric acid, ② EGFR, ③ serum creatinine, ④ serum urea nitrogen, and ⑤ adverse reactions.

### 2.2. Search Strategy

We searched PubMed, Embase, Cochrane Library, Web of Science, Wan-Fang database, China National Knowledge Infrastructure (CNKI), Chinese Scientific Journals Database (VIP), and CBM Libraries for relevant randomized controlled trials in each database from March 2012 up to March 2022. For English databases, we used free text terms such as “febuxostat” or “chronic kidney disease” or “hyperuricemia.” For the Chinese databases, it is suggested the search terms could be presented using the Chinese phonetic alphabet.

### 2.3. Literature Screening and Data Extraction

Two researchers conducted literature screening independently in strict accordance with inclusion and exclusion criteria. Then, they managed and identified the retrieved literature by the NoteExpress software (v.2.7.1). After picking, researchers read the topic and abstract for preliminary screening and then further read the full text for rescreening to determine whether to include and extract valid data, respectively, to establish Excel effective data extraction table. In case of disagreement, a third researcher shall be invited to solve the disagreement through consultation.

### 2.4. Statistical Analysis

The Stata 15.1 software was used to perform the meta-analysis. If for the binary classification variables using relative risk (RR), said the confidence interval (CI) is set to 95%. Continuity variables were represented by mean difference (MD), and confidence interval (CI) was set at 95%. Heterogeneity of research results was tested by *I*^2^. If *I*^2^ ≤ 50%, outcome data of fixed effects model (FE) were selected for analysis; if *I*^2^ > 50%, outcome data of random effects model (RE) were selected for reference analysis. At the same time, sensitivity analysis was used to observe heterogeneous sources and evaluate the stability of meta-analysis results.

## 3. Results

### 3.1. Search Results

Based on the search strategy, 631 references were identified. After excluding duplicate studies, 306 studies were scanned based on abstract and title. Then, 12 articles were evaluated in full text. After full text evaluation, 2 records were excluded for the following reasons: data mismatch (*n* = 1) and missing data (*n* = 1). Ultimately, 10 studies [13–16] were included in this meta-analysis (Table 1). The PRISMA statement flow chart shows this process (Figure 1).

### 3.2. Serum Uric Acid

Six studies reported the serum uric acid of the test group and the control group. Meta-analysis showed that the serum uric acid of the test group was significantly lower (SMD: -146.44, 95% Cl: -195.96, -86.93, and *P* < 0.01, Figure 2) than the control group. The results of all these trials showed high heterogeneity, and thus, a sensitivity analysis was conducted (Figure 3). Compared with the control group, febuxostat significantly reduces the level of uric acid in patients with CKD.

### 3.3. EGFR

Six studies reported the EGFR of the test group and the control group. Meta-analysis showed that the EGFR of the test group was significantly higher (SMD: 3.21, 95% Cl: 1.17, 5.25, and *P* < 0.01, Figure 4) than the control group. Compared with the control group, febuxostat significantly improves the EGFR level in patients with CKD and HUA.

### 3.4. Serum Creatinine

Six studies reported the serum creatinine of the test group and the control group. Meta-analysis showed that the serum creatinine of the test group was significantly lower (SMD: -15.27, 95% Cl: -20.75, -9.79, and *P* < 0.01, Figure 5) than the control group.

### 3.5. Serum Urea Nitrogen

Seven studies reported the serum urea nitrogen of the test group and the control group. Meta-analysis showed that the serum urea nitrogen of the test group was significantly lower (SMD: -2.37, 95% Cl: -3.31, -1.61, and *P* < 0.01, Figure 6) than the control group.

### 3.6. Adverse Reactions

Seven studies reported the adverse reactions of the test group and the control group. Meta-analysis showed that there was no significant difference in the adverse reactions between the test group and the control group (OR: 0.74, 95% Cl: 0.32, 1.68, and *P* = 0.47, Figure 7).

## 4. Discussion

Uric acid nephropathy is also known as hyperuricemia nephropathy or gouty nephropathy, and the main pathological changes are the renal pathological changes caused by uric acid crystal deposition and inflammatory cell infiltration are mainly manifested as interstitial nephritis and impaired renal tubular function and structure [17]. According to its pathological changes and clinical manifestations, it is mainly divided into 3 types: chronic uric acid nephropathy, acute uric acid nephropathy, and uric acid nephrolithiasis.

Uric acid is produced by the metabolism of DNA and/or RNA in the body and serves as the final product of purine metabolism. The product is excreted. Since humans lack urate oxidase and cannot decompose it into soluble allantoin, they are prone to hyperuricemia. Uric acid mainly comes from two ways: internal and external, of which endogenous accounts for 80%, which is synthesized by nucleic acid decomposition and amino acid, phosphoribosyl, etc. Nucleic acid protein food is decomposed. Uric acid is mainly excreted by the kidneys and intestines, of which 75% is excreted through the kidneys, and the rest is excreted after being degraded by microorganisms in the intestines [15, 18–20].

A total of 10 literatures were included in this study, including 436 patients in the experimental group and 427 in the control group. Meta-analysis showed that patients with CKD with HUA who received febuxostat had lower serum uric acid compared with controls. Meta-analysis showed satisfactory serum uric acid level for the experimental group (SMD: -146.44, 95% Cl: -195.96, -86.9, and *P* < 0.01). Based on the results of the meta-analysis of EGFR, compared with the control group, febuxostat significantly improves the EGFR level in patients with CKD with HUA (SMD: 3.21, 95% Cl: 1.17, 5.25, and *P* < 0.01). For the results of the meta-analysis of urine creatinine and urea nitrogen, compared with the control group, febuxostat significantly reduces the level of urine creatinine and urea nitrogen in patients with CKD with HUA (SMD: -15.27, 95% Cl: -20.75, -9.79, and *P* < 0.01 and SMD: -2.37, 95% Cl: -3.31, -1.61, and *P* < 0.01). There was no statistical difference in adverse reactions between the control group and the observation group after treatment (OR: 0.74, 95% Cl: 0.32, 1.68, and *P* = 0.47).

This study also has certain limitations. First, 10 RCTs included 863 patients. The overall sample size is not very large. All RCTs were single-center. The lack of multicenter studies may affect the representativeness of the conclusions to some extent. Second, the small sample size is not sufficient to fully assess the safety of febuxostat or other drugs.

## 5. Conclusion

The results of this study suggest that febuxostat may be effective in patients with CKD with HUA, as evidenced by serum uric acid, creatinine, urea nitrogen, and EGFR. However, large sample, multicenter, low risk of bias clinical studies, as well as basic medical research, are needed.

## Figures and Tables

**Figure 1:** Flow chart.

**Figure 2:** Forest illustration of the serum uric acid.

**Figure 3:** Sensitivity analysis of the serum uric acid.

**Figure 4:** Forest illustration of the EGFR.

**Figure 5:** Forest illustration of the serum creatinine.

**Figure 6:** Forest illustration of the serum urea nitrogen.

**Figure 7:** Forest illustration of the adverse reactions.

**Table 1:** Baseline characteristics.

Study (ref.)	Sample size (*T*/*C*)	Man/woman	Age (years) (mean ± SD) (*T*/*C*)	*T*	*C*	Outcomes
Huang 2018 [14]	42/41	27/14	61.97 ± 3.12	Febuxostat	Placebo	①③④⑤
Sircar 2015 [15]	45/48	66/27	56.22 ± 9.83/61.83 ± 12.00	Febuxostat	Placebo	②⑤
Zhang 2021 (1) [16]	36/30	41/25	80.13 ± 9.67	Febuxostat	Placebo	①②③④⑤
Zhao 2021 [17]	41/41	47/35	68.45 ± 5.20/68.56 ± 5.29	Febuxostat	Placebo	①③④⑤
Sezai 2015 [18]	56/53	85/24	69.4 ± 10.0/69.1 ± 9.2	Febuxostat	Allopurinol	②
Tanaka 2015 [19]	21/19	35/5	70.1 ± 9.5/66.1 ± 7.0	Febuxostat	Allopurinol	②
Zhang 2021 (2) [20]	27/27	31/23	51.58 ± 1.45/51.56 ± 1.44	Febuxostat	Allopurinol	①③④⑤
Zhu 2018 [21]	32/32	NA	NA	Febuxostat	Allopurinol	①③④⑤
Zhang 2021 (3) [22]	67/67	66/68	55.1 ± 9.4/54.2 ± 8.4	Febuxostat	Allopurinol	①②③④⑤
Wang 2022 [23]	69/69	96/42	81.35 ± 2.52/81.40 ± 2.49	Febuxostat	Allopurinol	①②④⑤

①: serum uric acid; ②: EGFR; ③: serum creatinine; ④: serum urea nitrogen; ⑤: adverse reactions.

## Data Availability

The data could be obtained by contacting the corresponding author.
